The article "Structure of Trials Assessing Endovascular Embolization for Brain Arteriovenous Malformations: A Scoping Review" was published in 2025. Journal: Cureus.

# Structure of Trials Assessing Endovascular Embolization for Brain Arteriovenous Malformations: A Scoping Review

**DOI:** 10.7759/cureus.83197

**Published:** 2025-04-29

**Authors:** Andrew Bohner, Humza Qureshi, Sachin Mysore, Arjun Kumar, Manisha Koneru

**Affiliations:** 1 Neurosciences, Cooper Medical School of Rowan University, Camden, USA; 2 Neurointerventional Surgery, Cooper University Health Care, Camden, USA

**Keywords:** cerebral arteriovenous malformations, clinical trials, data collection, embolization, research design

## Abstract

Recent advancements in embolic agents and endovascular techniques have led to increased interest in exploring endovascular embolization as a viable treatment for brain arteriovenous malformations. Several trials have investigated the use of various embolic agents for the treatment of arteriovenous malformations (AVMs) endovascularly. However, the reporting outcomes and design elements in these studies are heterogeneous and include inclusion/exclusion criteria and evaluated endpoints. This scoping review synthesized common endpoints cited within embolic endovascular AVM trials for monitoring their safety and efficacy, with a commentary on common threads of focus in future trials for evaluating AVM treatment, including adapting designs to be on par with the pace of advancements in endovascular technologies.

## Introduction and background

Brain arteriovenous malformations (AVMs) are primarily congenital malformations of cerebral vasculature composed of abnormal shunts that convalesce into a nidus, bypassing the normal capillary network [1]. Brain AVMs occur at a rate of 1.12-1.34 per 100,000 person-years, and can present with a mosaic of symptoms, ranging from asymptomatic to hemorrhage and ischemia [2]. Traditionally, brain AVMs were treated with either microsurgery, conservative management, or stereotactic radiosurgery; more recently, endovascular embolization has been used to treat AVMs [3]. There has been mixed evidence regarding the safety and efficacy of each of these modalities, driving the pursuit of additional research re-evaluating these treatment approaches as the technological landscape evolves [4-7]. Additionally, recent advances in neurovascular embolic agents and endovascular techniques have increasingly positioned embolization to be a promising modality for treating neurovascular pathologies such as AVMs [8-14]. This has specifically led to an increase in AVM studies evaluating the potential of endovascular embolization as both a standalone and adjunct therapy [15]. However, these studies lack established common elements for evaluating embolization efficacy and safety. In this review, we aim to summarize the common design elements and outcomes for studies evaluating endovascular embolization for brain AVM treatment, as summarizing previous reporting standards may help inform the designs of future studies.

## Review

Methods

This scoping review was exempt from institutional review board approval, and data were reported in accordance with the Preferred Reporting Items for Systematic Review and Meta-Analyses (PRISMA) guidelines.

Clinicaltrials.gov was queried for prospective studies added to the database before or on December 24, 2024, per the following search strategy: “(Arteriovenous Malformations OR AVM OR Arteriovenous Malformation) AND Embolization.” Studies were screened by two independent reviewers for inclusion based on the following criteria: 1) evaluated brain AVMs and 2) evaluated endovascular embolization as an intervention in at least one study arm. Full-text review and data extraction were performed with two independent reviewers to ascertain the following data elements: number of patients included, maximum follow-up duration, study population, study inclusion/exclusion criteria, and study endpoints.

*Statistical Analysis*

The primary outcome was the proportion of factors shared across all AVM embolization studies. Categorical variables were summarized as frequencies; continuous variables were summarized as medians and interquartile ranges (IQR). Data analyses were conducted using JMP version 18.0.0 (JMP Statistical Discovery LLC, Cary, NC).

Results

Eight studies met the inclusion criteria (Table 1; Figure 1). The median total study size was 117 patients (IQR 85-212), and follow-up was generally for one year on average (Table 2). Most studies included either both adult and pediatric patients (50.0%) or just adult patients (37.5%) (Table 2).

**Table 1:** Included trials AVMs: arteriovenous malformations

National Clinical Trial Identifier Number	Study Title
NCT06479343 [16]	Efficacy and Safety of the Liquid Embolic System (Tonbridge) for Endovascular Treatment of Cerebrovascular Malformations
NCT05058482 [17]	Non-Adhesive Liquid Embolic System in the Embolization of Cerebral Arteriovenous Malformations
NCT03691870 [18]	Transvenous Approach for the Treatment of Cerebral Arteriovenous Malformations
NCT02378883 [19]	Apollo Onyx Delivery Microcatheter Post Market Safety Study
NCT02098252 [20]	Treatment of Brain AVMs (TOBAS) Study
NCT02085278 [21]	Safety of Apollo Micro Catheter in Pediatric Patients
NCT00857662 [22]	Study Comparing Onyx and TRUFILL in Brain Arteriovenous Malformation
NCT00389181 [23]	A Randomized Trial of Unruptured Brain AVMs

**Figure 1:** Flow diagram of included trials AVMs: arteriovenous malformations

**Table 2:** Trial design features AVMs: arteriovenous malformations, IQR: interquartile range

Study Features	n=8
Total Study Size, median (IQR)	117 (85-212)
Maximum Duration of Follow-Up (months), median (IQR)	12 (6-48)
Study Population, no. (%)	
Both Adult and Pediatric	4 (50.0%)
Adult Only	3 (37.5%)
Pediatric Only	1 (12.5%)
Embolic Agent Used, no. (%)	
Onyx Liquid Embolic (Medtronic, Kalamazoo, MI, USA)	4 (50.0%)
TRUFILL n-BCA Liquid Embolic (Cerenovus Inc, Miami, FL, USA)	2 (25.0%)
Not Specified	3 (37.5%)
Specific Inclusion Criteria, no. (%)	
Brain AVM (Non-Specific Term)	7 (87.5%)
Only Unruptured AVMs	1 (12.5%)
Specific Spetzler-Martin Grades	2 (25.0%)
Specific Lawton-Young Grades	0 (0%)
AVM is in a Specific Location of the Brain	2 (25.0%)
Size of Nidus	0 (0%)
Specific Exclusion Criteria, no. (%)	
Pregnancy	5 (62.5%)
Contraindications for Angiography/Renal Failure	3 (37.5%)
AVM is not an Endovascular Candidate (i.e., Hemorrhage)	7 (87.5%)
Specific Spetzler-Martin Grades	1 (12.5%)
Specific Lawton-Young Grades	0 (0%)
AVM is in a Specific Location of the Brain	1 (12.5%)
Size of Nidus	0 (0%)
AVM Treated Previously by Other Modality	4 (50.0%)
Study Endpoints, no. (%)	
Procedure-Related Adverse Events	7 (87.5%)
Stroke/Neurological Deficit	5 (62.5%)
Reduction or Resolution of AVM on Imaging	3 (37.5%)
Mortality	2 (25.0%)
Clinical Symptom Improvement	2 (25.0%)
Hospital Readmission	1 (12.5%)
Residual AVM	1 (12.5%)

The most common inclusion criterion was generally stating the inclusion of brain AVMs (87.5%), followed by the inclusion of brain AVMs of particular Spetzler-Martin grades (25.0%) and AVMs located in specific regions within the brain (25.0%) (Table 2). The most common exclusion criterion was having an AVM that was not appropriate for endovascular management (87.5%), including surgical candidates or hemorrhagic AVMs (Table 2). Other common exclusion criteria include: pregnancy (67.5%); AVMs previously treated by other modalities (50.0%); and contraindications for angiography (37.5%) (Table 2).

The most common endpoints evaluated in these studies were peri-procedural adverse events (87.5%) and a new stroke or neurological deficit during the follow-up period (62.5%) (Table 2). Evaluation of other endpoints of interest, including radiographic appearance, clinical symptoms, or mortality, varied widely across studies (Table 2).

Discussion

We summarized common factors of study design across studies evaluating endovascular embolization for brain AVMs. Commonly, studies followed patients for around one year, emphasizing capturing short and long-term post-treatment complications. Moreover, clinical symptoms of neurological worsening are closely evaluated as an outcome of interest. However, outcomes aimed at evaluating adequate treatment or resolution, such as radiographic resolution or reduction in clinical symptoms, are lacking in current studies. As it is of clinical relevance for these prospective studies to not only evaluate the safety but also the efficacy of these interventions for treating AVMs, future studies may consider incorporating more radiographic outcomes focused on assessing AVM obliteration.

Moreover, the inclusion and exclusion criteria for these studies are broad and vary widely. As suggested in observational studies, focused evaluations within the substrata of AVMs may yield different insights than those examining a broad AVM population [4-7,24,25]. Certain AVM features, such as specific Spezter-Martin grades, the presence of multiple feeders, hemorrhagic presentation, and AVM rupture, differentially modify the success rate of each treatment approach and are unequally prone to various complications [24,26,27]. Thus, including more specific inclusion criteria or planning robust post-hoc analyses adequately powered to evaluate potential risks and benefits of endovascular embolization, among other treatment approaches, in these smaller subcohorts is needed to ensure potential treatment benefit or risk is not masked by cohort heterogeneity.

Additionally, several new embolic agents and endovascular tools have debuted within the past few years; however, standard follow-up durations in AVM trials are often 12 months or longer [28]. The length of these studies, often lasting several years before analysis, can make testing and evaluation of newer devices cumbersome and prohibitive. Adaptive clinical trial design can prove to be a useful model to push forward on this front, as this design offers the ability to discontinue certain experimental arms and include new interventional arms following interim points of analysis, which can offer substantial advantages over the standard two-arm trial model [29,30]. This type of trial design is well-suited for studies of AVM treatment, as rapid incorporation of trial arms can help yield data on pace with the introduction of newer tools and approaches to treatment. That is, employing this approach to AVM embolization studies can also allow these studies to adapt and collect data on clinically meaningful complications in both short-term and long-term settings, while mirroring the pace of new technology and techniques in the field. Future prospective studies and randomized clinical trials may consider utilizing adaptive designs in conjunction with standardized clinical and radiographic endpoints for safety and efficacy to augment the applicability of data yielded from AVM treatment studies.

## Conclusions

Current studies of endovascular embolization for brain AVM treatment are widely heterogeneous. With a one-year follow-up on average, these studies currently emphasize evaluating the rates of complications or neurological worsening. Future studies may consider incorporating standardized approaches to assessing adequate radiographic resolution. Given the heterogeneity and complexity of AVMs, more targeted designs with more specific inclusion and exclusion criteria may help identify meaningful differences in outcomes based on AVM characteristics (e.g., rupture status, grading, feeders). Likewise, rapid innovation in the embolic agents and endovascular tools used for the management of AVMs further reinforces the need for clinical trials to adapt alongside emerging technologies to more effectively assess the safety and efficacy of novel interventions. These adaptations in trial design may improve the precision of findings and better inform clinical decision-making.
